The article "Effect of Multivoice Chorus on Interpersonal Communication Disorder" was retracted in 2023. Reasons: signs of a paper mill; suspected computer-generated content; unreliable results or conclusions; lack of ethics approval or compliance.

# Effect of Multivoice Chorus on Interpersonal Communication Disorder

**DOI:** 10.1155/2022/6124778

**Published:** 2022-07-09

**Authors:** Huiling Lei

**Affiliations:** Hunan First Normal University, Changsha City, Hunan Province, China 410205

## Abstract

**Objective:**

As a type of music therapy, multipart chorus does not have high requirements for participants, and the basic level can be high or low. For college students, it is more likely to participate. Exploring the effect of multivoice chorus intervention on college students' mental health can provide reference for school psychological correction work. This study uses multivoice chorus as a means, combined with certain group psychological counseling techniques, to try to explore a new model for improving the mental health of college students.

**Method:**

Fifty college students in prison were selected as subjects and randomly divided into the control group and experimental group. The multivoice chorus method was used to conduct an intervention test on the mental health of the college students in the experimental group, and the observation was carried out for 3 months. Before and after the intervention, the anxiety self-rating scale, the trust scale, the social avoidance and distress scale, the shyness scale, the UCLA loneliness scale, and the college student psychological test personality subtest were used for psychological testing and evaluation. *Results/Discussion*. College students can actively recognize and reflect on their own behavior, and objectively evaluate others. Through the cognition and management of emotions, college students can handle personal emotions well in interpersonal communication. In the later stage of multivoice chorus, they can help each other, establish a mutual assistance system, help each other, and discuss and learn interpersonal communication skills together, so that college students can learn good interpersonal communication experience and skills from others in various interactions, achieve self-help, and promote college students to work together. In the process of interfering with interpersonal communication disorder, simple psychological counseling has also improved the phenomenon of interpersonal communication disorder, but the experimental effect is far from the effect of the combination of music education and psychological counseling, and it is relatively unstable in the stability test. In the specific operation, in the purely psychological counseling process, college students with interpersonal barriers do not actively cooperate with the intervention, the operating atmosphere is relatively dull, and the teachers are time-consuming and labor-intensive during the psychological counseling process, but the results are minimal. The only effect is also worn out within a few weeks, and the stability is poor. It can be seen that music education has played a pivotal role as a medium in the intervention of interpersonal communication disorders, which can make the intervention process easier, more effective, and more stable.

The article "Effect of Multivoice Chorus on Interpersonal Communication Disorder" was retracted in 2023. Reasons: signs of a paper mill; suspected computer-generated content; unreliable results or conclusions; lack of ethics approval or compliance.

## 1. Introduction

The art of multivoice chorus can be traced back to European churches in the middle ages and has a history of more than a thousand years. From the original “school music” to military songs, from the way of collective singing of Christian hymns to today's chorus art form with strong national characteristics, chorus art has gradually become an artistic image with novel themes, rich contents, and vivid images, and is widely accepted [1, 2]. It is inseparable from the tireless efforts of generations of composers [3].

After entering the university campus, the young and energetic college students are active in thinking and have a strong thirst for knowledge. Under the credit system, the open and free university environment could have opened their hearts, accepted themselves, made more friends, and had a good atmosphere for interpersonal communication. However, poor physical and psychological quality, complex social environment, and improper family education will affect the interpersonal relationships of college students.

College students are in an important period of needing guidance and care, and their physical and mental health is closely related to the future of the motherland and the destiny of the nation. During the university period, college students are in a critical period of going into society. The need for interpersonal communication is urgent, but there are many deficiencies in physical and mental development. High and favored by employers, good interpersonal relationships are the direct determining factor.

The influence of music on psychology is mainly manifested in the control and regulation of emotions [4]. Music directly acts on the human hypothalamic limbic system and other centers that manage emotions, and has a two-way regulating effect on human emotions [5]. When individuals are hit by reality or traumatized, they are particularly prone to strong emotional reactions such as anxiety and pain. Music can help people avoid traumatic situations or events, relieve depression and fear, and gradually return to normal. However, if the negative emotions are not fully released and regulated in time after being severely traumatized, the long-term repression of painful emotions in the heart can easily lead to the emergence of psychological posttraumatic sequelae [6, 7]. Music promotes the central system to regulate people's emotional activities, mobilize various factors such as memory, association, and imagination of people's thinking, arouse empathy, generate emotional resonance, and cause emotional reactions [8–10]. Therefore, music can release and vent the subject's emotions, turn negative emotions into positive ones, and transform excited emotions into peace or soothing, relieve physical stress, eliminate mental tension, and change people's emotions [11–13].

The article "Effect of Multivoice Chorus on Interpersonal Communication Disorder" was retracted in 2023. Reasons: signs of a paper mill; suspected computer-generated content; unreliable results or conclusions; lack of ethics approval or compliance.

This paper formulates and designs a multivoice chorus intervention program and implements it. Judging from the research results, the experiment has achieved the expected effect; from the subjective experience of the members of the experimental group and the observation of the therapist, the content of the activity has been recognized, and everyone is satisfied with the content and form of the experimental activity. There is a lot to gain from participating in multivoice chorus activities. Therefore, the plan of activity design has laid a practical foundation for further promotion of music group therapy by means of chorus in the school system.

Through the intervention of this multivoice chorus, the students in the experimental group relaxed their minds and body, relieved their psychological pressure, and prompted them to gradually understand themselves, understand themselves, improve themselves, and improve their adaptability; through interactive activities, they understand others more comprehensively, care for others, tolerate others, and establish a correct view of making friends. This research has improved the mental health level of the college students participating in the experiment as a whole and promoted the development of the mental health of the college students.

Through the development of the music therapy activities of the entire multivoice chorus group, the feedback of the members of the experimental group, and the observation of the therapist, the author believes that the use of the multivoice chorus music therapy method to intervene in the mental health of college students is effective.

This paper starts with the attribution of interpersonal communication disorder of college students, rationally analyzes the current application status of interpersonal communication disorder, and makes bold assumptions about music education as the main way of psychological intervention. This paper deeply explores the specific content and form of the combination of music education and psychological counseling, and demonstrates the application value and important role of music education in relieving college students' interpersonal barriers.

## 2. Methods

### 2.1. The General Idea of the Research

Fifty college students who were suitable for the experimental research conditions were selected from a university and randomly divided into the experimental group and the control group. Multivoice chorus method was used to intervene the mental health status of college students in the experimental group. The intervention duration was 3 months, 3 times a week, 30 minutes each time. College students in the control group did not receive any intervention. To explore whether multi part chorus can improve their mental health.

The article "Effect of Multivoice Chorus on Interpersonal Communication Disorder" was retracted in 2023. Reasons: signs of a paper mill; suspected computer-generated content; unreliable results or conclusions; lack of ethics approval or compliance.

### 2.2. The Formulation of the Plan

#### 2.2.1. Research Objects and Sampling

A school was selected, and 50 college students who met the following entry criteria were surveyed using the scale. The inclusion criteria are as follows: (1) age ≤ 50 years old, (2) able to read and understand the test questionnaire, (3) enrollment ≥ half a year, and (4) have normal language and communication skills and no mental disorder. A total of 50 questionnaires were distributed, and 50 valid questionnaires were recovered. According to the indicators of anxiety, low self-esteem, fluctuation, and other indicators in the test, combined with the results of other evaluations by the police, 50 college students were selected as the subjects and randomly divided into the experimental group and the control group with 25 students in each group. The difference was not statistically significant (all *P* > 0.05).

#### 2.2.2. Research Procedures

All the subjects filled out the “Anxiety Self-rating Scale”, “Trust Scale”, “Social Avoidance and Distress Scale”, “Shyness Scale”, “UCLA Loneliness Scale”, and “China Scales such as the Personality Sub-Test of College Students' Psychological Test” are required to be completed within 2 hours and taken back on the spot, and the results are used as the pretest data for the intervention.

The experimental group received multipart chorus intervention, 3 times a week, 50 minutes each time, and the duration was 3 months. The control group received no intervention.

Except for one subject who fell off due to illness, all the other subjects filled out the “Anxiety Self-rating Scale”, “Trust Scale”, “Social Avoidance and Distress Scale”, “UCLA Loneliness Scale”, “Chinese College Students' Psychological Test Personality Subtest”, and other scales, which are required to be completed within 2 hours and collected on the spot, and the results are used as the posttest data of the intervention.

For the statistics and processing of data, we use SPSS 19.0 software for statistical analysis of data.

#### 2.2.3. Selection of Research Tools

The Self-Rating Anxiety Scale (SAS) has 20 items and uses a 4-point scale to assess subjective feelings of anxiety. The cut-off value of the SAS standard score is 50 points, of which 50-59 is considered mild anxiety, 60-69 is moderate anxiety, and 70 or more is severe anxiety.

The article "Effect of Multivoice Chorus on Interpersonal Communication Disorder" was retracted in 2023. Reasons: signs of a paper mill; suspected computer-generated content; unreliable results or conclusions; lack of ethics approval or compliance.

The trust scale has 18 items and uses a 7-point score to measure the mutual trust of people with close relationships. It involves three connotations of trust: predictability (P), dependence (D), and trust (F). Predictability refers to whether we can predict the specific behavior of our peers, and dependability is the core component of trust. On the other hand, this “allows people to have unreserved confidence that their peers will continue to take responsibility and care for themselves.” The internal consistency coefficient for the entire scale was 0.83.

The Social Avoidance and Distress Scale consists of 28 items, of which 14 assess social avoidance and 14 assess social distress. The evaluation is on a 5-point scale. It measures the tendency to avoid social interaction and feelings of immersive distress. The internal consistency coefficient of the scale was 0.91, and the test-retest reliability was 0.69.

The Shyness Scale has 13 items. A 5-point scale is used, with higher scores indicating greater shyness. The internal consistency coefficient of the scale was 0.90, and the test-retest reliability was 0.89.

The UCLA Loneliness Scale has 20 items. A 4-point scoring system was used to evaluate loneliness due to the gap between the desire for social interaction and the actual level. The internal consistency coefficient of the scale was 0.94, and the test-retest reliability was 0.76.

### 2.3. Intervention Content and Its Operation

#### 2.3.1. Activity Venue and Equipment

The chorus activities are held in the multifunctional activity room of the school. The room is spacious and bright, with sufficient light and suitable temperature, which is conducive to maintaining a pleasant mood.

Equipment includes music CDs, multimedia computers, electronic keyboards, projectors, and stereos.

#### 2.3.2. Design Content of Multipart Chorus Intervention

The multivoice chorus method was used to intervene the mental health status of college students in the experimental group. The intervention test was completed by 3 full-time psychological counselors and 1 vocal music instructor from the Mental Health Guidance Center. The intervention duration was 3 months, 3 times a week, 50 minutes each time. College students in the control group did not receive any intervention.

Descriptive analysis was carried out on the psychological test results of the experimental group and control group before and after the intervention. The psychological test results of the same college student before and after the intervention were paired, and a paired *t*-test was carried out, and the difference between the psychological test results of the experimental group and the control group before and after the intervention was completely randomized. A *t*-test was designed. Data statistics use SPSS software.

The article "Effect of Multivoice Chorus on Interpersonal Communication Disorder" was retracted in 2023. Reasons: signs of a paper mill; suspected computer-generated content; unreliable results or conclusions; lack of ethics approval or compliance.

#### 2.3.3. Process Stages of Multivoice Chorus Intervention

In the early stage of the intervention, multivoice vocalization practice (5 to 10 minutes) and introduction to multivoice chorus-related knowledge and chorus skills requirements, organizing college students to enjoy chorus performances such as “My Motherland” and “Heavenly Road”, learn to sing the song “Farewell”.

In the middle stage of the intervention, multipart vocal practice (3 to 5 minutes), and chorus song practice, the main songs include “Road to Rejuvenation”, “Grateful Heart”, and “Let's Swing Double Pulp”.

For the later stage of the intervention, multivoice vocalization practice (about 3 minutes), and chorus song practice, the songs mainly include “Listening to Mom's Story of the Past” and “On the Taihang Mountains”; under the organization of the psychological counselor, each group of 10 people divided into 3 groups for discussion (1 time a week, 1.2 hours each time, 5 times in total), sharing the emotional experience of individual college students during the chorus.

#### 2.3.4. The Main Content of Multipart Chorus Activities

Before each singing activity, use games, rhythm, and other methods to achieve the purpose of enlivening the atmosphere, narrowing the distance, and paving the way for the next theme activities. The methods used in this series of activities in this study mainly include music relaxation, music rhythm body rhythm, music group interactive rhythm, music mini-games, and vocal practice.

According to the needs of the stage of intervention and the process of the activity, different levels of singing repertoire are used, and the corresponding activity content is designed according to the goals to be achieved in each activity. The methods used in this series of activities mainly include rhythm vocal practice, appreciation of excellent chorus repertoire, and practice of chorus repertoire.

After each activity, college students share their subjective experiences in the activity and express their own experiences and feelings, so as to express empathy, support each other, and grow together, which is also the core of each intervention process. Psychotherapists will actively encourage team members to speak up, discover, analyze, and solve problems through their own strengths and grow from the team.

Before the end of each activity, the therapist made a summary of the intervention activity and the performance of the college students in a timely manner, so that the college students could determine whether the activity achieved the expected goal. It is necessary to end the activity with encouraging words, and it is necessary to preset the introduction for the next activity, so as to keep the activity attractive to college students.

The article "Effect of Multivoice Chorus on Interpersonal Communication Disorder" was retracted in 2023. Reasons: signs of a paper mill; suspected computer-generated content; unreliable results or conclusions; lack of ethics approval or compliance.

## 3. Results

### 3.1. Evaluation of the Interpersonal Process

The evaluation of the interpersonal communication process can be based on the feedback of the multivoice chorus members participating in the multivoice chorus each time. After the unit sharing session, the multivoice chorus organizer will distribute the “Multi-voice Chorus Feedback Form” to 50 people in turn. The following is the score record of college students' feedback on activities in multivoice chorus, as shown in Figure 1.

The college students gradually accepted the multivoice chorus and expressed their approval and satisfaction with the activities and the leading methods designed by the multivoice chorus organizers. In the 6-phase multivoice chorus, the atmosphere was gradually harmonious, the interaction and communication among college students increased significantly, and the group motivation to support and encourage college students can play a role in positive energy guidance. In the end, the goal of multivoice chorus was basically achieved.

### 3.2. Evaluation of Multipart Chorus Effect

The effectiveness of polyphonic chorus in solving interpersonal communication problems of college students was evaluated by using the polyphonic chorus effect scale, in which 1 means agree, 2 means agree, 3 means average, 4 means disagree, and 5 means disagree.  Table 1 is the feedback of college students after the 6-period multivoice chorus.

From the results, the effect of interpersonal relationship growth activities is widely recognized by college students. Most college students can objectively recognize themselves, evaluate others, relieve emotional distress, learn interpersonal communication skills, and try to establish harmonious interpersonal relationships. The overall goal is basically achieved.

### 3.3. Self-Assessment of Multipart Chorus Organizers

During the preparatory period for the multivoice chorus work, the organizers found problems based on personal interviews and designed multivoice chorus according to the actual needs of college students' interpersonal communication and their growth characteristics. Multivoice chorus organizers do their job well, guide multivoice chorus members to learn and experience interpersonal relationships, accompany multivoice chorus members to grow, and coordinate the relationship between college students. During the whole process, the work attitude and principles of multivoice chorus organizers were recognized by college students.

The article "Effect of Multivoice Chorus on Interpersonal Communication Disorder" was retracted in 2023. Reasons: signs of a paper mill; suspected computer-generated content; unreliable results or conclusions; lack of ethics approval or compliance.

The organizers of multivoice chorus are constantly innovating the form and content of multivoice chorus during the activities. The indoor and outdoor multivoice chorus is combined to increase the fun and attract college students to continue to participate.

The organizers of the multivoice chorus did not make adequate preparations in advance and did not simply practice the process of interpersonal communication, resulting in the completion of the two multivoice choruses overtime.

Contribute to the problem-solving of college students, pass on their interpersonal experience to college students, and help them improve their interpersonal skills.

Multivoice chorus organizers focus on listening to the ideas and opinions of college students and giving appropriate feedback in a timely manner.

In short, the organizers of multivoice chorus follow the professional ethical values of social work and treat college students with respect, equality, and sincerity. The voice and autonomy of college students should be respected, the principles of self-determination and nonjudgment should be respected, and appropriate guidance should be given to the realization of the goal of multivoice chorus.

By carrying out six multivoice choruses with different goals, the college students are guided to learn from each other, comprehend with their hearts, and deeply experience and discuss together, so as to alleviate the loneliness and helplessness of college students. College students should play the role of “helping others and help themselves”, help each other, learn interpersonal communication skills together, gradually promote the achievement of the ultimate goal, improve interpersonal communication skills, and overcome interpersonal communication barriers.

### 3.4. Comparison between the Control Group and the Experimental Group

Figures 2 and 3 show the comparison of the results of the self-rating mental health scale SCL-90 in the control group before and after psychological counseling. According to SCL-90 evaluation, after psychological counseling, the improvement effect of the students in the control group was average, and the interpersonal relationship was improved significantly, *P* < 0.05. Among them, factors 1-9 are somatization, obsessive-compulsive state, interpersonal sensitivity, depression, anxiety, hostility, terror, paranoia, and psychosis.

Figures 4 and 5 show the comparison of the results of the self-rating mental health scale (SCL-90) before and after music education and psychological counseling in the experimental group. In the SCL-90 evaluation, due to the addition of music education in the experiment, the effects of obsessive-compulsive state, interpersonal sensitivity, depression, anxiety, hostility, terror, paranoia, and psychosis among the college students in the experimental group were very significant. Among them, the effect of interpersonal sensitivity and paranoia is extremely significant.

The article "Effect of Multivoice Chorus on Interpersonal Communication Disorder" was retracted in 2023. Reasons: signs of a paper mill; suspected computer-generated content; unreliable results or conclusions; lack of ethics approval or compliance.

### 3.5. Comparison of Stability Evaluation between the Control Group and Experimental Group

After the experiment, the stability test was compared, and the psychological health self-rating scale SCL-90 was evaluated and compared two weeks after the psychological counseling in the control group, as shown in Table 2. Table 2 shows that after two weeks of psychological counseling, the evaluation effect of the college students in the control group was not obvious and only slightly more effective in interpersonal sensitivity and depression than before the experiment, indicating that relying only on psychological counseling to alleviate the phenomenon of interpersonal communication barriers is unstable. Two weeks after the end of music education and psychological counseling in the experimental group, the self-rating scale of mental health SCL-90 was evaluated and compared, as shown in Table 3. It shows that after two weeks of music education and psychological counseling, the effect of the test on the college students in the experimental group is obvious. The effects of obsessive-compulsive state, interpersonal sensitivity, depression, anxiety, terror, paranoia, and psychotic factors are very significant among the college students in the experimental group. The hostile effect is extremely significant. Adding music education to the psychological counseling of college students with interpersonal communication disorder has a better and stable effect.

In short, after observing the subjects for a period of time, the members of the experimental group have less time to surf the Internet than the members of the control group, and they often participate in a series of cultural and sports activities in their daily life and study and communicate more smoothly with others. Teachers reported that some members of the experimental group had a high attendance rate in class and actively communicated with teachers about their learning status and completed their homework on time. The members of the control group performed better after the end of the experiment, but they did not last for a long time. The counselor reported that the members of the control group needed to talk and encourage each time to improve their daily routine and reduce their time online. The members of the experimental group will take the initiative to propose some music courses, such as learning tap dance, learning guitar, and learning music knowledge. They generally think that they are more and more interested in music and hope to improve themselves through music, promote the integration of arts and science, and improve their skills.

The article "Effect of Multivoice Chorus on Interpersonal Communication Disorder" was retracted in 2023. Reasons: signs of a paper mill; suspected computer-generated content; unreliable results or conclusions; lack of ethics approval or compliance.

## 4. Discussion

### 4.1. The Aesthetic Psychological Characteristics of College Students' Multivoice Music

Music aesthetic psychology refers to the individual's psychological state and mental ability in music aesthetic activities. It is the sum of musical feeling, musical perception, musical thinking, musical emotion, and personality characteristics [14]. Along with the different changes and characteristics of adolescents' physical and psychological development, their multivoice music aesthetic psychology will also show corresponding characteristics [15, 16].

#### 4.1.1. Multivoice Music Perception

Music is the art of hearing, and the ability to perceive and distinguish music is obtained through hearing at the same time. This perception includes the emotions expressed by the music, the overall perception of the music structure, the performance elements of the music, etc. In the multivoice chorus teaching of college students, in addition to rehearsal, listening and appreciation are also very important links [17–19]. In the process of listening and discrimination, college students can present a multidimensional effect through their ears on pitch, rhythm, beat, strength, interval, range, and timbre. At the same time, teachers should help college students build their sound perception ability in the process of listening and distinguishing, and pay attention to the details of music sound [20–22]. The cultivation of these music perception abilities is essential in chorus teaching [23].

With the growth of age, the accumulation of music experience and knowledge, college students have a clear motivation for learning. With the support of interest, music attention can last for a long time, and the amount of music content, the time of music memory, and the retention of music memory are greatly improved.

At this time, teachers should ask college students to make independent inspections and evaluations of their own chorus effects, and put forward their own perception comments on the works, so as to establish a sense of space by grasping the multivoice sound, so as to deepen the musical memory.

#### 4.1.2. Multipart Musical Thinking and Musical Imagination

The musical thinking of individual adolescents is creative, independent, general, and critical [9, 24]. In learning, they can look at problems comprehensively and can draw inferences from one case to the conclusion of a certain problem and draw parallels. Therefore, in the chorus teaching of college students, it should not be limited to the stage of emotional and pleasant appreciation, but also pay attention to the analysis from the aspects of melody, beat, rhythm, musical structure, and style. Traditional music in China has been linear since ancient times, and multivoice music has only been accepted and created since modern times. There is still a long way to go for the establishment and cultivation of multivoice musical thinking among today's young people [25–27]. Therefore, in teaching, in addition to appreciating and rehearsing multivoice works, teachers should also appropriately explain music theory, musical form, harmony, and other musical knowledge, so as to establish a rational understanding of polyphonic thinking [11, 28, 29].

The article "Effect of Multivoice Chorus on Interpersonal Communication Disorder" was retracted in 2023. Reasons: signs of a paper mill; suspected computer-generated content; unreliable results or conclusions; lack of ethics approval or compliance.

On the basis of rich music experience and knowledge, college students' imagination content is richer and gradually has the characteristics of creative imagination. Therefore, teachers should not instill one-sidedly in the course of teaching, but should give college students a broader space for their musical imagination, let the college students add harmony to the melody and listen to their own small pieces of works, increase the interest of college students, and enrich the music knowledge of college students.

#### 4.1.3. Cultivation of Interest in Multipart Music

The emotional development of music in adolescents is affected by the characteristics of their physiological development, and the changes in emotional activities are rich and intense [30–32]. With the growth and development of young people's bodies, the improvement of cognitive level, the active thinking, and the enhancement of self-awareness and adult consciousness, they are often infected and attracted by excellent music works, and resonate with the works [33]. At this time, teachers not only need to explain the expressiveness of musical works but also enable college students to comprehensively understand the knowledge of multivoice music, the background of the works, the life of the composer, and the expressive style of the era in which the works are located [34].

Music interest is one of the conditions for music learning. A lasting and stable interest in music will drive individuals to participate in music learning and music activities, and achieve good results. Adolescence is a critical period for establishing interest in music; especially in adolescence, individuals are still in a semimature state psychologically [35]. At this time, it is very important to guide the establishment of interest in multivoice music. Because the age of college students is in a sensitive stage, the artistic treatment of songs should be conducted by mutual discussion between teachers and students, and a variety of comprehensive methods should be used in the performance of songs. In terms of rehearsal methods, teaching content, music selection, etc., it is necessary to use rich and flexible teaching methods and choose beautiful music that conform to the aesthetic tastes of today's young people, and choreography methods such as singing and dancing, so that college students can establish a good relationship with each other [36].

The article "Effect of Multivoice Chorus on Interpersonal Communication Disorder" was retracted in 2023. Reasons: signs of a paper mill; suspected computer-generated content; unreliable results or conclusions; lack of ethics approval or compliance.

### 4.2. Discussion on Multivoice Chorus and Humanistic Quality Education

#### 4.2.1. The Establishment of Collective Consciousness

In the chorus, “unity” and “sameness” are very important principles, and this “unity” and “sameness” require everyone to tolerate, coordinate, and accommodate each other, which is conducive to training teenagers' collective consciousness and unity consciousness [37]. The unity of chorus has been incorporated into the category of social education.

In chorus, according to the needs of the acoustic effects presented by multiple voices, individual voices and individual singers need to judge the voices of those around them, judge the voices of their own voices, and more importantly, judge the voices of the entire chorus group. And it seems abrupt, and it cannot only “silence” to reduce the strength of the entire voice, but also pay attention to the timbre and intonation not to break the balance of the entire group because of itself.

In the family environment and social environment of the only child in modern cities, children have strong self-consciousness and relatively weak collective consciousness. Therefore, it is more necessary to cultivate the cooperative spirit of college students, and chorus is just a favorable way to build collective consciousness.

#### 4.2.2. Comprehensive Improvement of Musical Literacy

Music literacy is a comprehensive quality education for learning music, including comprehensive theoretical education in reading scores, sight-singing, listening, rhythm, harmony, writing, music appreciation, and music history. In the training process of multivoice chorus, it is precisely to integrate this theoretical knowledge into classroom rehearsal, which is a powerful means to improve musical literacy [38, 39].

At present, music education for teenagers is mostly aimed at personal achievement. Children start to participate in various music enlightenment courses when they are 3 years old, start to learn a musical instrument in elementary school, and participate in various grades and competitions. However, why is it difficult for teenagers who are based on certain musical training to execute the conductor's instructions harmoniously and uniformly in the orchestra? This is because Chinese children's personal achievement music education focuses too much on the training of individual performance skills and lacks the process and experience of collaboration. In Western countries, there has been a tradition of sending children to choirs hundreds of years ago. The popularization of multivoice chorus education should be the key to improving the current youth music education.

The article "Effect of Multivoice Chorus on Interpersonal Communication Disorder" was retracted in 2023. Reasons: signs of a paper mill; suspected computer-generated content; unreliable results or conclusions; lack of ethics approval or compliance.

### 4.3. Discussion on Attribution Bias

Attribution refers to the process of pointing out the nature of the behavior or inferring its cause through the analysis of the behavior of others or oneself [22, 40]. It is the cognition of the behavior and the analysis of the cause. When college students encounter interpersonal barriers, they usually either seek help from the school, consult psychological counselors, seek ways to resolve the barriers, or summarize the reasons for their interpersonal barriers and take targeted measures to alleviate their problems. However, there are often more or less attribution biases in this process, resulting in the interpersonal barriers of college students not being resolved in time, or even getting worse, leading to mental health problems and affecting the study and life of college students [41].

Although many universities have counseling agencies and professional psychological teachers who specialize in solving psychological problems and interpersonal concerns of college students, due to the relaxed learning environment in universities, college students have much less learning pressure than high school, and they have more free time [42]. Words are no longer absolute authority. At the same time, college students are in the psychological weaning period, and their emotions are rich and strong, but they are also extremely unstable. College students yearn for maturity and independence and hope to be respected and understood. They may have a rebellious mentality for too much discipline and may have a distrustful attitude towards something unfamiliar with psychological counseling [43].

### 4.4. Discussion on Correct Attribution

To analyze and recognize the causes, consequences of college students' interpersonal communication barriers and the choice tendency of follow-up behaviors avoid attribution bias and advocate benign positive attribution among college students, which is conducive to helping them establish good interpersonal relationships. Therefore, guiding college students to make positive attributions plays a positive role in improving college students' interpersonal communication status, establishing college students' confidence in establishing good interpersonal relationships, and improving their enthusiasm for interpersonal communication [44].

The article "Effect of Multivoice Chorus on Interpersonal Communication Disorder" was retracted in 2023. Reasons: signs of a paper mill; suspected computer-generated content; unreliable results or conclusions; lack of ethics approval or compliance.

This kind of negative psychology will greatly weaken the self-confidence of college students in their interpersonal skills, cause college students to have psychological obstacles, and even lead to mental health problems and even autism and other psychological diseases in college students [45].

The school should create a good interpersonal communication environment for college students who have interpersonal barriers. For example, arrange some expert lectures to teach interpersonal skills, enrich the extracurricular knowledge of interpersonal communication for college students, and help college students improve their interpersonal skills; at the same time, encourage the class as a unit and often hold some small gatherings or gatherings, to create opportunities for students to understand each other and reduce misunderstandings and interpersonal friction between students.

A file should be established for the mental health and interpersonal status of college students, which should be specially managed by psychological counselors, and the current situation of college students should be updated frequently to facilitate timely detection of problems.

College students themselves should also correctly understand themselves, recognize that everyone has their own advantages, do not have to be too inferior, participate in more collective activities and public welfare undertakings, and actively integrate into the university collective.

### 4.5. Deepen Empowerment Intervention and Expand Solutions

There are various modes of weighting, and different modes can be selected according to different objects. In college campuses, the use of empowerment intervention to help college students resolve interpersonal barriers can be achieved by considering the empowerment at the individual level and the empowerment at the school level [46].

Empowerment at the individual level is primarily for individuals. For those college students who have interpersonal barriers, they often have self-denial or self-dwarfing psychology because of interpersonal problems. They are largely passive recipients of interpersonal relationships, their own ability to empower is weak, and it is difficult to make changes on their own to adapt themselves to the interpersonal atmosphere of the school [47]. Therefore, professional school counselors are needed to mobilize the enthusiasm of college students with communication barriers, help them discover their abilities, enable them to control their mood and communication skills, and enable them to better integrate into campus life and establish good interpersonal relationships. The main purpose of empowering individuals is to develop the ability to adapt to the surrounding environment and to express their needs under various conditions [17, 48]. Therefore, schools can help college students to correct their psychological biases by means of psychological counseling and education, so that they have the opportunity to reevaluate themselves and use this to analyze the reasons for their failure or weakness and the opportunities to develop themselves [14, 25, 49].

The article "Effect of Multivoice Chorus on Interpersonal Communication Disorder" was retracted in 2023. Reasons: signs of a paper mill; suspected computer-generated content; unreliable results or conclusions; lack of ethics approval or compliance.

In order to reduce the alienation, isolation, and sense of powerlessness of college students with interpersonal barriers, members of peer groups in the same situation can be encouraged to establish mutual aid groups and to get rid of the sense of powerlessness through the awakening of collective consciousness and joint efforts. The intervention of multivoice chorus is beneficial to eliminate the loneliness, self-centeredness, and selfishness of these college students and enhance the mediating role of the social support system in alleviating the plight of college students with interpersonal barriers.

The development of multivoice chorus has created a good interpersonal communication environment for college students with interpersonal communication barriers, increased their chances of successful interpersonal communication, enriched their successful experience, and improved their confidence in interpersonal interaction.

## 5. Conclusion

Multivoice chorus organizers organize this group to promote their interaction, communication, and sharing through multivoice chorus and guide them to establish a mutual aid system and gain support. The organizers of multivoice chorus focus on college students as the main body, focus on the common problems faced by college students, and under the guidance of professional values, use the form of multivoice chorus to let college freshmen relax and relieve stress in multivoice chorus. At the same time, it guides college students to interact, communicate, express emotions, solve problems together, improve interpersonal skills, and overcome interpersonal barriers during the entire multivoice chorus process. Therefore, to solve the problem of college students' interpersonal communication barriers, it is the best way to carry out multivoice chorus. The intervention of multivoice chorus can effectively help college students improve their interpersonal skills, overcome interpersonal barriers, establish harmonious interpersonal relationships, and adapt to new life more quickly, thereby promoting their physical and mental health. The results of the study show that with simple basic music education courses combined with corresponding music performance activities and appreciation activities, people with interpersonal communication disorders not only participated in the music experience but also received physical and mental relaxation exercises, appropriately vented their suppressed emotions, and found in the music activities. The intervention of interpersonal barriers of college students has opened up a new way, and it has played a unique educational value in the psychological health education consulting work in colleges and universities. Music education is added to the psychological counseling of college students with interpersonal communication barriers. The experiment shows that music education can alleviate the phenomenon of interpersonal communication barriers and some psychological problems of college students.

The article "Effect of Multivoice Chorus on Interpersonal Communication Disorder" was retracted in 2023. Reasons: signs of a paper mill; suspected computer-generated content; unreliable results or conclusions; lack of ethics approval or compliance.

## Figures and Tables

**Figure 1:** Score statistics of multivoice chorus feedback.

**Figure 2:** Comparison of SCL-90 assessment results before and after psychological counseling.

**Figure 3:** Comparison of *t* value and *P* value of SCL-90 assessment results before and after psychological counseling.

**Figure 4:** Comparison of SCL-90 assessment results before and after music education and psychological counseling.

**Figure 5:** Comparison of *t* value and *P* value of SCL-90 assessment results before and after music education and psychological counseling.

**Table 1:** Statistics of self-assessment of multivoice chorus effect.

Project	Ability to objectively recognize oneself and evaluate others	Willingness to trust and understand others	Can relieve interpersonal emotional distress and can control and manage emotions	Learn interpersonal communication skills (listening, praise, appropriate feedback, polite rejection, etc.)	Willing to take the initiative to communicate with people and establish harmonious interpersonal relationships	Know how to grasp the scale of interpersonal communication
Agree	33	41	39	36	38	42
Relatively agree	6	4	5	8	12	5
Generally	4	2	4	3	0	2
Rather disagree	5	2	1	1	0	1
Disagree	2	1	1	2	0	0

**Table 2:** Comparison of SCL-90 stability evaluation results before and after psychological counseling.

Factor	Somatization	Obsessive state	Interpersonal sensitivity	Depression	Anxiety	Hostility	Fear	Paranoia	Psychosis
Before therapy	1.8	2.6	2.4	1.8	1.6	2.1	2.3	2.1	1.8
After treatment	1.6	2.4	2.5	1.7	1.9	1.8	2.1	1.7	2.3
*t*	1.5	1.9	1.7	1.6	2	2.4	2.6	1.9	2.2
*P*	0.14	0.03	0.02	0.01	0.03	0.03	0.01	0.02	0.01

**Table 3:** Comparison of SCL-90 assessment results before and after music education and psychological counseling stability.

Factor	Somatization	Obsessive state	Interpersonal sensitivity	Depression	Anxiety	Hostility	Fear	Paranoia	Psychosis
Before therapy	1.8	2.6	2.4	1.8	1.6	2.1	2.3	2.1	1.8
After treatment	1.2	2.1	2.2	1.4	1.1	1.7	2.0	1.5	2.0
*t*	1.9	2.9	2.6	1.9	2.8	2.9	3.2	2.9	2.8
*P*	0.04	0.02	0.01	0.01	0.02	0.01	0.00	0.00	0.00

The article "Effect of Multivoice Chorus on Interpersonal Communication Disorder" was retracted in 2023. Reasons: signs of a paper mill; suspected computer-generated content; unreliable results or conclusions; lack of ethics approval or compliance.

## Data Availability

The data used to support the findings of this study are included within the article.

## References

[1] Zhang L.-K., Sun S.-Q., Xing B.-X., Luo R.-M., Zhang K.-J. (2019). Using psychophysiological measures to recognize personal music emotional experience. *Frontiers of Information Technology & Electronic Engineering*.

[2] Sturm B. L., Ben-Tal O., Monaghan Ú. (2019). Machine learning research that matters for music creation: a case study. *Journal of New Music Research*.

[3] Doi S., Sakanno A., Muto T., Sakano Y. (2017). Reliability and validity of a Japanese version of the valuing questionnaire (VQ). *Japanese Journal of Behavior Therapy*.

[4] Maia A., Oliveira J., Lajnef M. (2019). Oxidative and nitrosative stress markers in obsessive–compulsive disorder: a systematic review and meta-analysis. *Acta Psychiatrica Scandinavica*.

[5] Hughes L. S., Clark J., Colclough J. A., Dale E., McMillan D. (2017). Acceptance and commitment therapy (ACT) for chronic pain. *The Clinical Journal of Pain*.

[6] MacRae A. (2021). The influences of inter music therapy on music therapists who experience it. *Nordic Journal of Music Therapy*.

[7] Soleimani V., Sahebkar A., Hosseinzadeh H. (2018). Turmeric (Curcuma longa) and its major constituent (curcumin) as nontoxic and safe substances: review. *Phytotherapy Research*.

[8] Skoro M., Roncevic A. (2019). The music industry in the context of digitization. *Economic and Social Development*.

[9] Shima T., Kawai T., Yanagihara M., Kumano H. (2016). Validation of the Japanese version of the cognitive fusion questionnaire: the 13-item content revised version and the 7-item version. *Japanese Journal of Behavior Therapy*.

[10] Zhao Y., Wang Z., Shan J. (2017). On the importance of music therapy to college students’ mental health. *Forum on Industry and Technology*.

[11] Shawky R., Kamal T. M., Raafat S., el Nady G. H. (2018). Genotyping of PPAR-*γ* gene polymorphism in Egyptian neonates affected with sepsis disease and its severity. *Egyptian Journal of Medical Human Genetics*.

[12] Mardomingo Sanz M. J., Sancho Mateo C., Soler López B. (2019). Assessment of comorbidity and social anxiety in adolescents with attention deficit hyperactivity disorder: the SELFIE study. *Anales de Pediatría*.

[13] Oliveira A. I., Pinho C., Fonte P., Sarmento B., Dias A. C. P. (2018). Development, characterization, antioxidant and hepatoprotective properties of poly(Ɛ-caprolactone) nanoparticles loaded with a neuroprotective fraction of Hypericum perforatum. *International Journal of Biological Macromolecules*.

The article "Effect of Multivoice Chorus on Interpersonal Communication Disorder" was retracted in 2023. Reasons: signs of a paper mill; suspected computer-generated content; unreliable results or conclusions; lack of ethics approval or compliance.

[14] Xiao C. (2019). Research on the advantages of music therapy intervention for college students’ mental health. *Northern Music*.

[15] Gulbins A., Grassmé H., Hoehn R. (2016). Regulation of neuronal stem cell proliferation in the hippocampus by endothelial ceramide. *Cellular Physiology and Biochemistry*.

[16] Jang B. Y., Heo W. H., Kim J. H., Kwon O. W. (2019). Music detection from broadcast contents using convolutional neural networks with a Mel-scale kernel. *EURASIP Journal on Audio, Speech, and Music Processing*.

[17] Hollocks M. J., Lerh J. W., Magiati I., Meiser-Stedman R., Brugha T. S. (2019). Anxiety and depression in adults with autism spectrum disorder: a systematic review and meta-analysis. *Psychological Medicine*.

[18] Meng J. (2019). Feasibility analysis of music therapy in the development of college students’ mental health education. *Curriculum Education Research*.

[19] Zukerman G., Yahav G., Ben-Itzchak E. (2019). Increased psychiatric symptoms in university students with autism spectrum disorder are associated with reduced adaptive behavior. *Psychiatry Research*.

[20] Birajdar G. K., Patil M. D. (2019). Speech and music classification using spectrogram based statistical descriptors and extreme learning machine. *Multimedia Tools and Applications*.

[21] Rutter K. J., Ashraf I., Cordingley L., Rhodes L. E. (2020). Quality of life and psychological impact in the photodermatoses: a systematic review. *The British Journal of Dermatology*.

[22] Brander G., Pérez-Vigil A., Larsson H., Mataix-Cols D. (2016). Systematic review of environmental risk factors for obsessive-compulsive disorder: a proposed roadmap from association to causation. *Neuroscience and Biobehavioral Reviews*.

[23] Ahn M. Y., Ham S. A., Yoo T. (2018). Ligand-activated peroxisome proliferator-activated receptor *δ* attenuates vascular oxidative stress by inhibiting thrombospondin-1 expression. *Journal of Vascular Research*.

[24] Hiller J., Belt C., Gardstrom S., Willenbrink-Conte J. (2021). Safeguarding curricular self-experiences in undergraduate music therapy education and training. *Music Therapy Perspectives*.

[25] Zou H. (2018). The application of music therapy in college students’ mental health education. *Journal of Jilin Institute of Chemical Technology*.

[26] Rosen T. E., Mazefsky C. A., Vasa R. A., Lerner M. D. (2018). Co-occurring psychiatric conditions in autism spectrum disorder. *International Review of Psychiatry*.

[27] Bai Z., Luo S., Zhang L., Wu S., Chi I. (2020). Acceptance and commitment therapy (ACT) to reduce depression: a systematic review and meta-analysis. *Journal of Affective Disorders*.

The article "Effect of Multivoice Chorus on Interpersonal Communication Disorder" was retracted in 2023. Reasons: signs of a paper mill; suspected computer-generated content; unreliable results or conclusions; lack of ethics approval or compliance.

[28] Panda R., Malheiro R., Paiva R. P. (2020). Novel audio features for music emotion recognition. *IEEE Transactions on Affective Computing*.

[29] Kar S. K., Choudhury I. (2016). An empirical review on oxidative stress markers and their relevance in obsessive-compulsive disorder. *International Journal of Nutrition Pharmacology Neurological Diseases*.

[30] Sarkar R., Choudhury S., Dutta S., Roy A., Saha S. K. (2020). Recognition of emotion in music based on deep convolutional neural network. *Multimedia Tools and Applications*.

[31] Anastopoulos A. D., DuPaul G. J., Weyandt L. L. (2018). Rates and patterns of comorbidity among first-year college students with ADHD. *Journal of Clinical Child and Adolescent Psychology*.

[32] McLeod J. D., Meanwell E., Hawbaker A. (2019). The experiences of college students on the autism spectrum: a comparison to their neurotypical peers. *Journal of Autism and Developmental Disorders*.

[33] Farrokhmanesh M., Hamzeh A. (2019). Music classification as a new approach for malware detection. *Journal of Computer Virology and Hacking Techniques*.

[34] Cuffe S. P., Visser S. N., Holbrook J. R. (2020). ADHD and psychiatric comorbidity: functional outcomes in a school-based sample of children. *Journal of Attention Disorders*.

[35] Nelson J. M., Liebel S. W. (2018). Anxiety and depression among college students with attention-deficit/hyperactivity disorder (ADHD): cross-informant, sex, and subtype differences. *Journal of American College Health*.

[36] Khoramnia S., Bavafa A., Jaberghaderi N. (2020). The effectiveness of acceptance and commitment therapy for social anxiety disorder: a randomized clinical trial. *Trends in Psychiatry and Psychotherapy*.

[37] del Casale A., Sorice S., Padovano A. (2019). Psychopharmacological treatment of obsessive-compulsive disorder (OCD). *Current Neuropharmacology*.

[38] Mosner M. G., Kinard J. L., Shah J. S. (2019). Rates of co-occurring psychiatric disorders in autism spectrum disorder using the Mini International Neuropsychiatric Interview. *Journal of Autism and Developmental Disorders*.

[39] Spain D., Sin J., Linder K. B., McMahon J., Happé F. (2018). Social anxiety in autism spectrum disorder: a systematic review. *Research in Autism Spectrum Disorders*.

[40] Kato T. A., Kanba S., Teo A. R. (2019). Hikikomori: multidimensional understanding, assessment, and future international perspectives. *Psychiatry and Clinical Neurosciences*.

[41] Veale D., Gledhill L. J., Christodoulou P., Hodsoll J. (2016). Body dysmorphic disorder in different settings: a systematic review and estimated weighted prevalence. *Body Image*.

The article "Effect of Multivoice Chorus on Interpersonal Communication Disorder" was retracted in 2023. Reasons: signs of a paper mill; suspected computer-generated content; unreliable results or conclusions; lack of ethics approval or compliance.

[42] Koelsch S., Vuust P., Friston K. (2019). Predictive processes and the peculiar case of music. *Trends in Cognitive Sciences*.

[43] Chen F., Yu X., Meng G. (2019). Hippocampal genetic knockdown of PPAR*δ* causes depression-like behaviors and neurogenesis suppression. *The International Journal of Neuropsychopharmacology*.

[44] Napoli E., Siracusa L., Ruberto G. (2018). Phytochemical profiles, phototoxic and antioxidant properties of eleven Hypericum species-a comparative study. *Phytochemistry*.

[45] Zhu H., Liu Q., Yuan N. J., Zhang K., Zhou G., Chen E. (2020). Pop music generation. *ACM Transactions on Knowledge Discovery from Data*.

[46] Miller M. L., Brock R. L. (2017). The effect of trauma on the severity of obsessive-compulsive spectrum symptoms: a meta-analysis. *Journal of Anxiety Disorders*.

[47] Eleazu C. O. (2016). Characterization of the natural products in cocoyam (Colocasia esculenta) using GC–MS. *Pharmaceutical Biology*.

[48] Ding N., Patel A. D., Chen L., Butler H., Luo C., Poeppel D. (2017). Temporal modulations in speech and music. *Neuroscience & Biobehavioral Reviews*.

[49] Li X. (2018). Analysis of the effectiveness of music therapy on college students’ mental health. *Contemporary Music*.

